The article "Image Classification in HTP Test Based on Convolutional Neural Network Model" was published in 2021. Journal: Comput Intell Neurosci.

# Image Classification in HTP Test Based on Convolutional Neural Network Model

**DOI:** 10.1155/2021/6370509

**Published:** 2021-10-08

**Authors:** Lin Liu

**Affiliations:** School of Art and Design, Wuhan University of Technology, Wuhan, Hubei 430070, China

## Abstract

HTP test in psychometrics is a widely studied and applied psychological assessment technique. HTP test is a kind of projection test, which refers to the free expression of painting itself and its creativity. Therefore, the form of group psychological counselling is widely used in mental health education. Compared with traditional neural networks, deep learning networks have deeper and more network layers and can learn more complex processing functions. In this stage, image recognition technology can be used as an assistant of human vision. People can quickly get the information in the picture through retrieval. For example, you can take a picture of an object that is difficult to describe and quickly search the content related to it. Convolutional neural network, which is widely used in the image classification task of computer vision, can automatically complete feature learning on the data without manual feature extraction. Compared with the traditional test, the test can reflect the painting characteristics of different groups. After quantitative scoring, it has good reliability and validity. It has high application value in psychological evaluation, especially in the diagnosis of mental diseases. This paper focuses on the subjectivity of HTP evaluation. Convolutional neural network is a mature technology in deep learning. The traditional HTP assessment process relies on the experience of researchers to extract painting features and classification.

## 1. Introduction

In recent years, artificial intelligence can be widely used in deep learning of complex patterns and multiple scenes and has made a series of major breakthroughs in the fields of image recognition and speech recognition [1]. HTP (House Tree Person) test in psychometrics is a widely studied and applied psychological assessment technique. HTP test can also be used as an intelligence evaluation test, which is mainly based on the evaluation of painting details. The traditional test is a psychological projection test, which can be effectively applied to psychological diagnosis, treatment, and related research. The test can reflect the painting characteristics of different groups, has good reliability and validity after quantitative scoring, and has high application value in psychological evaluation, especially in the diagnosis of mental diseases. HTP test is a kind of projection test, which refers to the free expression of painting itself and its creativity. It is a test form that awakens the different manifestations of the inner world or personality characteristics of the examinee, so as to project their inner needs and desires in the process of painting [2]. According to statistics, nearly 85% of human's access to external information comes from images. With the rapid development of computer Internet, communication, software, and hardware technology, human beings have entered an era of information explosion [3]. People pay more and more attention to the expression and processing of image information. The process of image classification and recognition includes image preprocessing, image segmentation, key feature extraction, and matching recognition. With the help of the latest image classification technology, we can not only obtain the required information faster for image retrieval but also apply it to scientific experiments, traffic recognition, safety protection, medical devices, face recognition, and other fields [4].

The article "Image Classification in HTP Test Based on Convolutional Neural Network Model" was published in 2021. Journal: Comput Intell Neurosci.

The essence of psychology lies in exploring the mysteries of human beings. Therefore, psychologists try to use various tools to understand human beings [5]. Faced with the contradiction that the number of people with psychological problems is increasing and the strength of psychological counselling is obviously insufficient, it is difficult for individual counselling to ensure that everyone can get counselling in time and effectively. Therefore, the form of group psychological counselling is widely used in mental health education [6]. Compared with traditional neural networks, deep learning networks have deeper and more network layers and can learn more complex processing functions. Pictures bring us a convenient way to record and share information, but it is difficult for us to use the information expressed by images. More and more companies and researchers use deep learning to discuss and study image classification, which provides a good development for artificial intelligence [7]. Convolution neural network, a deep learning technology widely used in image classification task of computer vision, can automatically complete feature learning on data without manual feature extraction [8]. The image is mapped from low-level features to high-level features through multiple hidden layers, and the classification task is completed under the function of the classifier.

In the era of rapid development of information technology, it is the trend of the times to let computers replace human beings to deal with a large amount of information and solve the cognitive limitations of human beings [9]. Conforming to the trend of the times and responding to the policy call, convolution neural network, a new technology in artificial intelligence, is applied to HTP test in psychological measurement field. At this stage, image recognition technology can be used as an aid to human vision. People can quickly get the information in pictures by searching [10]. For example, you can take a picture of an object that is difficult to describe and quickly search for the related content. Compared with the existing convolution neural network, convolution neural network will be more reasonable and efficient, with less training time, more reasonable data results, and other advantages, and make it achieve higher accuracy than the existing technology in the application of image classification [11]. We mainly summarize and comment on the basic principle of HTP, its application in various fields of psychological counselling, and the existing problems, in order to promote its further promotion and application in China [12].

The article "Image Classification in HTP Test Based on Convolutional Neural Network Model" was published in 2021. Journal: Comput Intell Neurosci.

The innovative contribution of this paper is to apply convolution neural network technology to psychometrics. Convolutional neural network has developed rapidly in recent years and has achieved good results in the fields of natural language, image, speech recognition, video, and so on. Among HTP modules and tree modules, export-oriented, stable, and social modules are the main choices. The main block is an inward, stable, and gregarious mold. Each can reflect the personality, vitality, and self of the family.

## 2. Related Works

In the field of psychology and clinical application research, subjects are given pencil, rubber, and white paper, and they are required to draw on white paper. The evaluators analyze and evaluate the painting content according to certain standards, so as to understand the psychological phenomenon, intelligence state, personality, and other content of the subjects. Cai and Guo put forward the painting characteristics of shadow and repeated description to reflect the anxiety of the subjects and thought that the expression of shadow or black anxiety was common in neurosis, obsessive-compulsive personality, and other mental patients [13]. Liu et al. developed a computer-aided analysis system for HTP based on a large number of clinical studies. The computer-aided system is a summary of experts' experience, which uses computers to store records, and tries to standardize the processing of painting image information with the help of computers. At present, there are also commercial psychological evaluation companies in the market that have developed similar computer-aided systems for HTP tests [14]. Liu et al. propose that the HTP test, as a nonverbal diagnostic method, can effectively reflect depression that cannot be expressed in words [15]. Li et al. establish a logistic regression model for the pathological symptoms and personality traits of painters and their related painting characteristics and predict and judge the psychological state and personality traits by using painting characteristics [16].

The article "Image Classification in HTP Test Based on Convolutional Neural Network Model" was published in 2021. Journal: Comput Intell Neurosci.

Cheng and Zhang put forward the conclusion that the painting features of middle school students in suicide plan are more likely to have many houses, moon and sharp parts of the picture, less people with open mouth, and sun, and the window is relatively small [17]. These forms of painting characteristics have a certain reference value for the evaluation of middle school students' suicide problem. Backpropagation (BP) algorithm was proposed in [18]. This algorithm solves the XOR problem of perceptron and reduces the computational complexity of the neural network. It has been widely used in various fields and has set off the climax of neural network research. Yu et al. studied the HTP of 137 nonclinical community adults and 121 clinical patients and their social introversion subscale of Minnesota multiple personality test and found that there was no significant difference between the two groups [19]. Huang et al. divide 273 primary school students into normal and abnormal groups by applying Children Somatization Scale and Achenbach Child Behavior Scale and make regression analysis according to the characteristics of HTP test. The results showed that there were significant differences in the frequency of 12 painting features between the somatization group and the normal group [20]. Tang et al. put forward neuron model, describe the formal mathematical description of neurons and the method of network structure, and verify that a single neuron has logic function, thus opening the door of artificial neural network [21]. Gao et al. conducted Cartel Sixteen Personality Tests and HTP Tests on medical students and found that there were significant differences in painting characteristics such as pen strength, painting symmetry, lines, and tree types. Painting test is a kind of projection test, which is based on psychodynamics, and allows the subjects to express their psychological state and activities hidden in the subconscious without restriction [22].

## 3. HTP Drawing Test

### 3.1. HTP Drawing Test Theory

The word “projection” was first proposed by Freud, which belongs to the psychological defense mechanism. Translated: it is the psychological tendency of individuals to unconsciously reflect their thoughts, attitudes, wishes, emotions, personality, and other psychological characteristics in the interpretation of things [23]. People's defense psychology against painting is low, and subconscious information (such as motivation, emotion, anxiety, conflict, and values) can be projected in paintings [24]. They do not have a certain meaning in themselves, but the reactions they cause are of special significance. The meaning comes from the subjective explanation and thought of the test stimulus. Unconsciously, it projects its psychological needs, personality, emotion, motivation, conflict, defense, and other internal states. Among the various painting tests, the HTP test is the most classic one, which is composed of three familiar elements: room, tree, and human [25].

The article "Image Classification in HTP Test Based on Convolutional Neural Network Model" was published in 2021. Journal: Comput Intell Neurosci.

HTP test not only has auxiliary value for evaluating emotional states such as anxiety and depression but also has reference significance for stress states. Using the HTP test to evaluate personality can avoid direct vocabulary from attacking and avoiding special subjects. Avoid sensitive words causing their bad emotions or reactions. The HTP projection test focuses on the evaluation of subconsciousness and has the function of intervention and guidance. It has a broad application prospect in mental health education. The combination of house, tree, and human can not only greatly reduce the burden of the subjects but also more effectively detect the personality characteristics of the subjects, improve the success rate, and expand the test objects, as shown in Figure 1.

At present, the measurement of personality is mainly self-report scale, and these psychological tests are all conducted by asking subjects to give positive or negative answers to questions. Subjects tend to answer questions according to the values generally accepted by society and conceal their true thoughts. The HTP test is mainly based on the psychodynamic point of view, which holds that houses, as places where people live, can cause associations with families and relatives. The pictures of trees can reflect the subjects' unconsciousness. People reflect the subjects' self-image and the situation of getting along with others. There are differences in psychological development between autistic children and normal children. HTP test can reflect the specific aspects of the differences. In China, the HTP painting test is still in the early stage of development. In view of its unique advantages, it has great research value and application space.

### 3.2. HTP Drawing Test Research Summary

At present, there are two main research orientations of painting test: meaning interpretation orientation and painting feature analysis orientation. The former analyzes the meaning of painting and the psychological state or personality of the painter. The latter establishes the connection between the psychological state of painting expression and personality traits by establishing standardized evaluation criteria of painting characteristics and combining with the self-report scale. First of all, the psychological test of painting is not limited by language, cognitive ability, and age. It can accommodate more information such as subjects' mental state, cognition of their own roles, and interaction with the environment and others. Secondly, according to psychoanalytic theory, people's subconscious or defense mechanism always resists exploring the inner world out of the need of protecting individuals. However, college students generally lack of self-awareness and largely rely on the evaluation of others. Therefore, the nonverbal nature of HTP can well reflect the hidden personality traits and help individuals to realize themselves. The HTP drawing test analyzes a case of family counselling on mother-daughter communication problems. The results show that through the process of painting and analysis, the communication between mother and daughter is improved, and the effect of family counselling is better.

The article "Image Classification in HTP Test Based on Convolutional Neural Network Model" was published in 2021. Journal: Comput Intell Neurosci.

## 4. Convolutional Neural Network

### 4.1. The Architecture of Convolutional Neural Networks

Convolutional neural network is a model in deep learning. The typical convolution network structure is that many researchers improve the structure and performance of convolution network and improve the universality of network and the accuracy of image recognition and classification, as shown in Figure 2.

Neural network is a computing model composed of a large number of neural units connected with each other. The MNIST database is constructed by NIST's SD-1 and SD-3 databases and contains a series of binary handwritten digital images. The NIST database uses SD-3 database as the training sample set and SD-1 as the test sample set. SD-3 is clearer and easier to identify than SD-1. SD-3 database is collected from handwriting of staff of census bureau, and SD-1 is collected from students in high school. The test error of 60 iterations on MNIST database and cifar-10 database is reduced by using the optimization algorithm, as shown in Figures 3 and 4.

It can be seen from the experiment that SGD without driving quantity can gradually reduce the error, but the speed and effect of decline are average. The effect of SGD and NAG with driving capacity is better than that of SGD, but the gradient decreases slowly in the early stage and then gradually stabilizes, and the effect of SGD with driving capacity is better than that of NAG. ADAGRAD's descending speed is stable, so the curve is smooth and the effect is good.

After changing the amount of data and after 1000 steps of iteration, the experimental results on two databases are obtained, as shown in Figures 5 and 6.

The article "Image Classification in HTP Test Based on Convolutional Neural Network Model" was published in 2021. Journal: Comput Intell Neurosci.

In the process of training, it can be seen that, with the increase of the number of training on MNIST database and CIFAR-10 database, the test error will gradually decrease, and with the increase of data, it can effectively prevent overfitting.

These simple processing units constitute a large-scale parallel distributed processor, which can continuously acquire knowledge from the external environment through the learning process. That is, weights are used to store acquired knowledge, which is equivalent to the activation of a cell's memory by artificial neural networks. The neural cells in the visual cortex have very complex patterns, and they are very sensitive to the subregions in the visual region. These subregions are called local receptive fields, and all subregions can be tiled to cover the whole visual area. Traditional neural networks usually have only two or three layers of structure design, while deep networks have more layers and more functional layers. For example, the lower sampling layer is designed to achieve specific learning efficiency.

Convolutional neural network is a network structure often used in deep learning technology. Because of the short development period of deep learning, its application in image classification has been a research topic only recently one or two years. Therefore, image classification based on deep learning is a new and promising research topic. For the two analysis formulas *A* and *B* established by LFW face gender classification, a large number of matching schemes can be obtained through their relationship. The relationship between classification accuracy *a* and time complexity *B* is obtained on LFW dataset, and the abscissa and ordinate values of each solid point reflect the time complexity of the network under the current classification accuracy. When the classification accuracy begins to decline, the time complexity drops very quickly and then tends to be flat, as shown in Figure 7.

The learning methods all have a certain structure, and there are many hidden neural networks. Therefore, all machine learning methods with a hierarchical structure can be called deep learning. In fact, the predecessor of deep network is the traditional artificial neural network. The biggest difference between them is mainly reflected in the number of network layers and network complexity. It consists of simple cell layer, which is responsible for responding to specific stimuli in receptive field, extracting features, and alternating complex cell layer, which can be regarded as the first network implementation of convolutional neural network. Neural network reduces the number of network parameters by sharing weights and extracts the optimal local features by limiting the receptive field. Finally, we hope that the neural network can automatically achieve translation invariance, and all these functions can be implemented in a convolutional neural network.

The article "Image Classification in HTP Test Based on Convolutional Neural Network Model" was published in 2021. Journal: Comput Intell Neurosci.

### 4.2. Image Classification in Convolutional Neurovision

There are many ways for human beings to perceive external information, including hearing, sight, smell, taste, and touch. In other words, the purpose of data preprocessing is to reduce or even eliminate data redundancy. If a dataset contains many irrelevant samples or noisy redundant information, it is difficult to find them during the training phase. The number of free parameters of convolutional neural network is greatly reduced due to the way of local connection and neurons sharing weights. 55 groups of control parameters are randomly selected to form 55 different networks to train the model, and the error between the predicted value obtained by the precision analysis formula and the actual test value of the model is compared, as shown in Figure 8.

55 groups of control parameters are randomly selected to form 55 different network training models, and the errors between the predicted values obtained by the time complexity analysis formula and the time values used in the actual test of the models are compared, as shown in Figure 9.

The initial weight value and deviation value can be randomly sampled by a zero-mean Gaussian function. The function of this random initialization is to break the symmetry. In addition, the image feature translation, scaling, and distortion invariance of the pooling layer is very good. In addition, there are many good algorithms, but they are constantly prompted by the convolutional neural network. Convolutional neural network has a major breakthrough in image features, so it is more convenient. Therefore, the industry uses more convolutional neural networks.

Image classification is a technology that uses computers to process, analyze, and understand images in order to identify various targets and objects with different patterns and classifies images into one of several categories. It plays an important role in image-based data acquisition and processing. Generally speaking, the simpler the network and the smaller the configuration parameters in the network, the less time it takes to train the model and apply the test. Although the complex network is more time-consuming during training and testing and requires higher equipment, it will eventually show better performance. Specifically, for a single training example (*x*_*i*_, *y*_*i*_), a squared difference loss function can be defined as follows, where *f*_*W*,*b*_(*x*) is used to calculate the output value of the forward propagation and *W* and *b* represent the weight value and the bias value, respectively:

(1) $$\begin{array}{c} J\left(W,b;x_{i},y_{i}\right)=\frac{1}{2}{\left\|f_{W,b}\left(x_{i}\right)-y_{i}\right\|}^{2}. \end{array}$$

For all *m* training samples, the total loss function is defined as follows:

(2) $$\begin{array}{c} J\left(W,b\right)=\frac{1}{m}\sum_{i=1}^{m}J\left(W,b;x_{i},y_{i}\right),\\ J\left(W,b\right)=\frac{1}{m}\sum_{i=1}^{m}\left(\frac{1}{2}{\left\|f_{W,b}\left(x_{i}\right)-y_{i}\right\|}^{2}\right). \end{array}$$

In order to avoid overfitting, a regular term or weight attenuation term is usually added to the loss function. Weight decay is not used for bias terms. *W*_*ij*_^*l*^ is the weight value, where is the layer index and *ij* is the neuron index of the adjacent hidden layer. The weight attenuation parameter is *λ*, and the correlation between the square error term and the regularization term has been controlled. *λ* The larger the model is, the smaller the value of *W*_*ij*_^*l*^ is, which means that the model changes less and shows stronger generalization ability:

(3) $$\begin{array}{c} J\left(W.b\right)=\frac{1}{m}\sum_{i=1}^{m}\left(\frac{1}{2}{\left\|f_{W,b}\left(x_{i}\right)-y_{i}\right\|}^{2}\right)++\frac{\lambda }{2}\sum_{l=1}^{nl-1}\sum_{i=1}^{Sl}\sum_{j+1}^{Sl+1}{\left(W_{ij}^{l}\right)}^{2}. \end{array}$$

The purpose of training is the process of minimizing the loss function (*W*, *b*). This can be done by updating *w* and *b* by gradient descent. Parameters *w* and *b* are updated in a small range in each iteration of gradient descent. *α* indicates the learning rate that controls this range:

(4) $$\begin{array}{c} \Delta W_{ij}^{l}=\alpha \frac{\partial }{\partial W_{ij}^{l}}J\left(W,b\right),\\ \Delta b_{j}^{l}=\alpha \frac{\partial }{\partial b_{j}^{l}}J\left(W,b\right). \end{array}$$

The derivative of loss function *J*(*W*, *b*) with respect to weight and bias is defined as follows:

(5) $$\begin{array}{c} \frac{\partial }{\partial W_{ij}^{l}}J\left(W,b\right)=\frac{1}{m}\sum_{i=1}^{m}\frac{\partial }{\partial W_{ij}^{l}}J\left(W,b;x_{i},y_{i}\right)+\lambda W_{ij}^{l},\\ \frac{\partial }{\partial b_{i}^{l}}J\left(W,b\right)=\frac{1}{m}\sum_{i=1}^{m}\frac{\partial }{\partial b_{i}^{l}}J\left(W,b;x_{i},y_{i}\right)+\lambda W_{ij}^{l}. \end{array}$$

For neurons in each layer of the network, an error term can be used to represent the error between the output value and the real value.

The article "Image Classification in HTP Test Based on Convolutional Neural Network Model" was published in 2021. Journal: Comput Intell Neurosci.

Image classification methods are divided into two categories. The first category classifies images in image space domain or transform domain. The second is to use convolution neural network to learn image features automatically for image classification. First, change one of the controllable parameters while keeping the other parameters unchanged. The relationship between the classification accuracy *y* and the filter size *x* obtained on the CIFAR-10 data set is shown in Figure 10.

Convolutional neural network learns hierarchical feature description in a supervised or unsupervised way and directly uses image pixel information as input, as shown in Figure 11.

All the information of the input image is retained to the greatest extent. The feature extraction and high-level abstraction are carried out by convolution operation, and the model outputs the result of image recognition directly. Convolutional neural network has the ability to combine hierarchical features of images.

## 5. Conclusions

In this paper, convolution neural network technology is applied to psychometrics. Convolutional neural network has developed rapidly in recent years and achieved good results in natural language, image, speech recognition, video, and other fields. Convolution neural network model has learned the essential difference between HTP paintings drawn by normal and abnormal groups, that is to say, it relies on matrix operations such as convolution and pooling of network, instead of the task of summarizing and extracting painting features and then classifying and diagnosing painting images in a large number of practices. We are looking forward to the study of HTP standardization by domestic scholars in the future. Among HTP modules and tree modules, extroverted, stable, and gregarious modules are the main choices. The main block is an inward, stable, and gregarious mold. Each one can reflect the personality characteristics of family, vitality, and self. HTP can be tested separately or used for group counselling. Objective psychological test is widely used in clinic because of its high objective reliability and simple interpretation standard. Especially, in the screened interview, the HTP projection test is used as the interview medium to enable the subjects to explain HTP painting and quickly understand the subjects' inner conflict and feelings. This not only greatly improves the speed and accuracy of projection but also communicates with the subconscious and integrates itself through painting and uses its art therapy to promote the rehabilitation of mental patients. Although the final result has not completely reached the standard that can be applied to clinical diagnosis, however, we believe that the convolution neural network method is a new possibility for HTP mapping test evaluation, and it is also a new idea for psychometric research.

The article "Image Classification in HTP Test Based on Convolutional Neural Network Model" was published in 2021. Journal: Comput Intell Neurosci.

## Figures and Tables

**Figure 1:** HTP painting image.

**Figure 2:** Basic architecture of convolutional neural network.

**Figure 3:** Experimental results of different optimization algorithms on the MNIST database.

**Figure 4:** Experimental results of different optimization algorithms on the CIFAR-10 database.

**Figure 5:** Changes of errors on the MNIST database with data enhancement.

**Figure 6:** Changes of errors on the CIFAR-10 database with data enhancement.

**Figure 7:** Time complexity under LFW classification accuracy.

**Figure 8:** The error between the predicted value and the actual test value of the model.

**Figure 9:** The error between the predicted value and the actual test time value of the model.

**Figure 10:** The relationship between classification accuracy *y* and filter size *x*.

**Figure 11:** The structure of a convolutional neural network.

## Data Availability

The data used to support the findings of this study are available from the corresponding author upon request.

## References

[1] Zhou S., Shen W., Zeng D., Fang M., Wei Y., Zhang Z. (2016). Spatial-temporal convolutional neural networks for anomaly detection and localization in crowded scenes. *Signal Processing: Image Communication*.

[2] Chang Y., Yan L., Fang H., Zhong S., Liao W. (2019). HSI-DeNet: hyperspectral image restoration via convolutional neural network. *IEEE Transactions on Geoscience and Remote Sensing*.

[3] Sun Y., Lin Z., Guan W., Zhao F. (2017). Multi-input convolutional neural network for flower grading. *Journal of Electrical and Computer Engineering*.

[4] Gao W., Fang Y., Zhang F., Yang Z. (2020). Representation learning of knowledge graphs using convolutional neural networks. *Neural Network World*.

[5] Zhou S., Liang W., Li J., Kim J.-U. (2018). Improved VGG model for road traffic sign recognition. *Computers, Materials & Continua*.

[6] Alam M., Wang J. F., Cong G., Yunron L., Chen Y. (2021). Convolutional neural network for the semantic segmentation of remote sensing images. *Mobile Networks and Applications*.

[7] Dede M. A., Aptoula E., Genc Y. (2019). Deep network ensembles for aerial scene classification. *IEEE Geoscience and Remote Sensing Letters*.

[8] Xie J., He N., Fang L., Plaza A. (2019). Scale-free convolutional neural network for remote sensing scene classification. *IEEE Transactions on Geoscience and Remote Sensing*.

[9] Fukui H., Yamashita T., Yamauchi Y., Fujiyoshi H., Murase H. Pedestrian detection based on deep convolutional neural network with ensemble inference network.

[10] Zhang X., Wang Z., Liang L. (2018). A stacking algorithm for convolutional neural networks. *Computer Engineering*.

The article "Image Classification in HTP Test Based on Convolutional Neural Network Model" was published in 2021. Journal: Comput Intell Neurosci.

[11] Luo F., Wang P., Xu G., Lei Y., Fan Y. (2020). Anomaly prediction of crowd gathering based on multi-scale convolutional neural network. *Computer Engineering and Science*.

[12] Huang T., Hu B. (2020). Pedestrian attribute recognition based on lightweight convolutional neural network in surveillance scene. *Electronic measurement technology*.

[13] Cai L., Guo H. (2019). Population flow prediction based on convolutional neural network. *Computer and Information Technology*.

[14] Gardner P., Bull L. A., Gosliga J., Dervilis N., Worden K. (2021). Foundations of population-based SHM, part III: heterogeneous populations-mapping and transfer. *Mechanical Systems and Signal Processing*.

[15] Liu G., Jiang X., Tang B. (2021). Application research of feature selection and convolutional neural network in crop fine classification. *Journal of Geo-Information Science*.

[16] Nan L., Cai J., Li K. (2020). Convolutional neural network face recognition algorithm based on multiple inception structure. *Computer System Application*.

[17] Cheng H., Zhang C. (2019). Apple image recognition technology based on improved LeNet convolutional neural network in natural scenes. *Food and Machinery*.

[18] Liu Y. (2016). Evaluation of the application of HTP test in the general survey of psychological assessment of recruits. *South China National Defense Medical Journal*.

[19] Yu J., Luo L., Luo Y. (2016). Study on the rehabilitation of 50 patients with schizophrenia treated with integrated HTP painting. *Contemporary Nurse*.

[20] Carter C. K., Hartley C. (2021). Are children with autism more likely to retain object names when learning from colour photographs or black-and-white cartoons?. *Journal of Autism and Developmental Disorders*.

[21] Costa D. B., Bastos A. G., Schütz D. M. (2020). Personality and psychopathological aspects in animal hoarding measured through HTP. *Contextos Clínicos*.

[22] Gao Y., Zhou P., Qiao K. (2017). Professional achiever factors and HTP test for medical students. *Chinese Journal of Health Psychology*.

[23] Jeong S. Y., Lee Y. B., Jeong H., Kim K. O. (2020). A brief study of response patterns in the S-HTP test based on Sasang constitution. *Journal of Oriental Neuropsychiatry*.

[24] Liu T. (2017). A case study of the application of projective painting to the psychological supervisors of the adult viewing cases. *Counselling Quarterly*.

[25] Miao Li (2019). Investigation and research on the status quo of college students’ happiness——based on HTP projection psychology analysis. *Journal of Chizhou University*.

